This article has been retracted.

# Recombinant Human Adenovirus-p53 Injection Induced Apoptosis in Hepatocellular Carcinoma Cell Lines Mediated by p53-Fbxw7 Pathway, Which Controls c-Myc and Cyclin E

**DOI:** 10.1371/journal.pone.0068574

**Published:** 2013-07-01

**Authors:** Kangsheng Tu, Xin Zheng, Zhenyu Zhou, Chao Li, Jing Zhang, Jie Gao, Yingmin Yao, Qingguang Liu

**Affiliations:** Department of Hepatobiliary Surgery, First Affiliated Hospital of Medical College of Xi’an Jiaotong University, Xi’an, Shaanxi, China; University of Minnesota, United States of America

## Abstract

F-box and WD repeat domain-containing 7 (Fbxw7/hAgo/hCdc4/Fbw7) is a p53-dependent tumor suppressor and leads to ubiquitination-mediated suppression of several oncoproteins including c-Myc, cyclin E, Notch, c-Jun and others. Our previous study has indicated that low expression of Fbxw7 was negatively correlated with c-Myc, cyclin E and mutant-p53 in hepatocellular carcinoma (HCC) tissues. But the role and mechanisms of Fbxw7 in HCC are still unknown. Here, we investigated the function of Fbxw7 in HCC cell lines and the anti-tumor activity of recombinant human adenovirus-p53 injection (rAd-p53, Gendicine) administration *in vitro* and *in vivo*. Fbxw7-specific siRNA enhanced expression of c-Myc and cyclin E proteins and increased proliferation in cell culture. rAd-p53 inhibited tumor cell growth with Fbxw7 upregulation and c-Myc and cyclin E downregulation *in vitro* and a murine HCC model. This effect could be partially reverted using Fbxw7-specific siRNA. Here, we suggest that the activation of Fbxw7 by adenoviral delivery of p53 leads to increased proteasomal degradation of c-Myc and cyclin E enabling growth arrest and apoptosis. Addressing this pathway, we identified that rAd-p53 could be a potential therapeutic agent for HCC.

## Introduction

HCC is one of the most common malignancies worldwide. It is a common cancer and occurring with increasing frequency in China [1]. Ubiquitination by the ubiquitin-proteasome system (UPS) is a post-translational modification that regulates diverse cellular processes, including cell proliferation, cell cycle progression, transcription, immune response, DNA damage repair and apoptosis [2,3]. The UPS consists of the ubiquitin-activating enzyme (E1), the ubiquitin-conjugating enzyme (E2), and the ubiquitin-protein ligase (E3). Among the E3 ubiquitin ligase enzymes, the SKP1-CUL1-F-box (SCF) E3 ligase complex is one of the best characterized. Fbxw7 is a member of the F-box protein family, which determines the substrate specificity of the SCF-type E3 complex, and is able to target various oncogenic proteins for ubiquitination such as Cyclin E, c-Myc, c-Jun, Notch, Presenilin, Mcl-1, Sterol regulatory element-binding proteins (SREBP), mTOR, Krüppel-like factors (KLFs), c-Myb and Aurora A [4–6]. Because all these characterized substrates are well known oncogenic proteins that are frequently overexpressed in a variety of human cancers, Fbxw7 is believed to be a tumor suppressor that contributes to the negative regulation of these oncogenic proteins [6]. Our previous study has indicated that the mRNA and protein expression of Fbxw7 was significantly down-regulated in the HCC tumor tissues compared to the normal tumor-adjacent tissues. Fbxw7 protein was expressed at significantly lower levels in patients with high histological grade and advanced tumor-node-metastasis (TNM) stage [7]. But the role and mechanisms involved in Fbxw7 are still unclear in HCC.

p53 gene functions as the cellular gatekeeper for cell growth, division and induction of cell death through apoptosis, mutations and deletions of p53 gene are detectable in about 50% of HCCs [8]. In addition, loss of functional p53 gene is associated with poorly-differentiated HCCs, a shorter tumor-free interval and survival time [9,10]. Hence, reconstitution of a wild-type p53 gene is an attractive therapeutic approach to treat HCC. Fbxw7 has been identified as a p53 target gene [11,12]. In support of this notion, Fbxw7 was dramatically up-regulated by infection with adenovirus-mediated transfer of wild-type p53 into the p53-deficient cells [4]. Moreover, p53-binding sites were discovered in the Fbxw7 exon, further emphasizing Fbxw7 as a direct target of p53 [11]. Fbxw7 targets for ubiquitination and degradation of c-Myc and Cyclin E, cell cycle regulators that are frequently deregulated in HCC [13,14]. Our previous study pointed out that Fbxw7 protein expression was negatively correlated with c-Myc, Cyclin E and mutant-p53 in HCC tissues [7]. We hypothesize that deregulation or mutations in p53 contribute to hepatocarcinogenesis through Fbxw7, c-Myc and Cyclin E pathway.

In this report, we investigated the function of Fbxw7 in HCC, then treated HCC cells with rAd-p53 and evaluated p53, Fbxw7, c-Myc and Cyclin E expression and anti-tumor activities *in vitro* and *in vivo*. rAd-p53 is a gene therapy drug that is used to treat neck squamous cell carcinoma (HNSCC) [15]. It is composed of replication-incompetent adenovirus serotype 5 (Ad5) encoding for human wild-type p53 gene. Our results suggest that rAd-p53 administration induces HCC growth arrest and apoptosis by Fbxw7-dependent c-Myc and Cyclin E proteolysis.

## Materials and Methods

### Ethics statement

All animal protocols were approved by the Institutional Animal Care and Use Committee of Xi’an Jiaotong University (Permit Number: 2012-0096).

### Cell culture

The immortal human liver cell line LO2 and HCC cell lines SMMC-7721, HepG2, Hep3B, Huh7 and Bel-7402 were obtained from the Institute of Biochemistry and Cell Biology, Chinese Academy of Sciences (Shanghai, China). All the cells were maintained in Dulbecco’s modified Eagle medium (DMEM, Hyclone, USA) containing 10% fetal bovine serum (FBS, Gibco BRL, USA) with 100 units/mL penicillin and 100 µg/mL streptomycin (Sigma, USA) and cultured in a humidified 5% CO_2_ incubator at 37°C.

### *Fbxw7* sequence

The *Fbxw7* (α, β and γ) sequence was amplified using cDNA from LO2, SMMC-7721, HepG2, Hep3B, Huh7 and Bel-7402 cells with KOD-FX DNA polymerase (TOYOBO, Japan) and sequencing primers (Table 1). These PCR products were separated on 1% agarose gels containing ethidium bromide (EB) and purified with ethanol precipitation. Purified PCR products were sequenced by Shenzhen Huada Gene Technology Co., Ltd. (China).

**Table 1:** Primers for *Fbxw7* sequence and PCR amplification.

**Sequencing primers**	**5’–3’**
Fbxw7α-1F primer	ATGAATCAGGAACTGCTCTCTGTGGGC
Fbxw7α-1R primer	CTCAGAACCATGGTCCAACTTTCTTTTCA
Fbxw7α-2F primer	CATACACATACTAACAGTGTCACGAACTCCA
Fbxw7α-2R primer	CTCCAGTAGCGACATGTCTGAGCTGCT
Fbxw7α-3F primer	GATGCAAGTGATAGAACCCCAGTTTCAAC
Fbxw7α-3R primer	TCTCTGCATTCCACACTTTGAGTGTCC
Fbxw7α-4F primer	GTCTGAGAACATTAGTGGGACATACAGGT
Fbxw7α-4R primer	TCTTTGAGTTCCATTCCACTTGTTAACG
Fbxw7α-5F primer	TGATACATCAATCCGTGTTTGGGATGT
Fbxw7α-5R primer	TCACTTCATGTCCACATCAAAGTCCAG
Fbxw7β-1F primer	ATGTGTGTCCCGAGAAGCGGTTTGATACTG
Fbxw7β-1R primer	CTCAGAACCATGGTCCAACTTTCTTTTCA
Fbxw7γ-1F primer	ATGTCAAAACCGGGAAAACCTACTCTAAAC
Fbxw7γ-1R primer	CTCAGAACCATGGTCCAACTTTCTTTTCA
**PCR primers**	
Fbxw7-F primer	AAAGAGTTGTTAGCGGTTCTCG
Fbxw7-R primer	CCACATGGATACCATCAAACTG
p53-F primer	ATTCTGGGACAGCCAAGTC
p53-R primer	TAGTTGTAGTGGATGGTGGTA
c-Myc-F primer	CTTCTCTCCGTCCTCGGATTCT
c-Myc-R primer	GAAGGTGATCCAGACTCTGACCTT
Cyclin E-F primer	GTTATAAGGGAGACGGGGAG
Cyclin E-R primer	TGCTCTGCTTCTTACCGCTC
GAPDH-F primer	CAAGCTCATTTCCTGGTATGAC
GAPDH-R primer	CAGTGAGGGTCTCTCTCTTCCT

Reverse transcription-polymerase chain reaction (RT-PCR) and real-time quantitative RT-PCR (qRT-PCR)

Fbxw7-specific oligonucleotide primers were designed to amplify a 249-bp PCR product encoding the common region among three Fbxw7 isoforms. The primers in Table 1 were used for PCR. RT-PCR was performed as previous report [5]. PCR amplification for quantification of Fbxw7, c-Myc, Cyclin E and (glyceraldehyde-3-phosphate dehydrogenase) GAPDH mRNA was done in the ABI PRISM 7300 Sequence Detection System (Applied Biosystems, USA) using the SYBR® Premix Ex Taq^TM^ ii(Perfect Real Time) Kit (Takara Bio, Japan). Three experimental replicates were performed.

### Colony formation assay

200 LO2, SMMC-7721, HepG2, Hep3B, Huh7 and Bel-7402 cells were placed in a fresh six-well plate in triplicate and maintained in DMEM containing 10% FBS for 2 weeks. Cell colonies were fixed with 20% methanol and stained with 0.1% coomassie brilliant blue R250 at room temperature for 15 min. The colonies were counted by ELIspot Bioreader 5000 (BIO-SYS, Karben, GE).

### Fbxw7 RNA interference

Fbxw7-specific siRNA, sense 5-GGAGUAUGGUCAUCACAAAtt-3 and antisense 5-UUUGUGAUGACCAUACUCCac-3 (Silencer Predesigned siRNA, GenePharma Co. Ltd, Shanghai, China) and TurboFect Transfection Reagent (Thermo Scientific, USA) were then added in 6-well plates. After incubation, cells were seeded at 1.5x10^5^ per well in a volume of 2 mL in 6-well plates and incubated at 37°C and 5% CO_2_. The RNA interference assay was done after 24 h incubation.

### MTT Assay

Proliferation was determined using the 3-(4, 5-dimethylthiazol-2-yl)-2, 5-diphenyltetrazolium bromide (MTT) assay (Roche Diagnostics, USA). After 24 h incubation following Fbxw7-specific siRNA or rAd-p53 (Gendicine, Sibiono GeneTech Co., Ltd, Shenzhen, China) addition, cells were cultured further for 0 to 72 h and the absorbance of the samples was measured using a model 550 microplate reader (Bio-Rad Laboratories, CA, USA), at a wavelength of 570 nm corrected to 655 nm. Three experimental replicates were performed.

### Western blot analysis

Fbxw7 (ab74054, Abcam, Hong Kong) (1:1000), c-Myc (#5605, Cell Signaling Technology, Beverly, MA, USA) (1:1000), Cyclin E (#4129, Cell Signaling Technology, Beverly, MA, USA) (1:1000), p53 (S371, Bioworld Technology, St. Louis Park, MN, USA) (1:1000) and β-actin (sc-47778, SANTA CRUZ, CA, USA) (1:1000) antibodies were used for Western blot assay. Secondary horseradish peroxidase-conjugated goat anti-mouse or rabbit antibodies (Bio-Rad, USA) were used at a 1:5000 dilution and detected by the enhanced chemiluminescence reagent (Millipore, Billeria, MA, USA).

### Flow cytometry

An Annexin-V-FLUOS Staining Kit (Roche, USA) was used to analyze apoptosis levels. Briefly, Hep3B cells were infected by rAd-p53 for various times and 10^6^ treated cells were washed with PBS and centrifuged at 200×g for 5 min, then resuspended in 100µL of Annexin-V-FLUOS labeling solution (predilute 20 µL Annexin-V-Fluos labeling reagent in 1 mL Incubation buffer and add 20 µL Propidium iodide solution) and incubated 10-15 min at 15-25°C, the samples were analyze by BD FACS Canto II Flow Cytometer (Becton Dickinson, USA). Three experimental replicates were performed.

### *In vivo* treatments with rAd-p53

A nude mouse xenograft model was established using 4-6 week-old female BALB/c nude mice (Centre of Laboratory Animals, The Medical College of Xi’an Jiaotong University, Xi’an, China). Mice were housed in sterilized cage (2 animals/cage) with constant temperature and humidity and fed with regular autoclaved chow diet with water ad libitum. 10^7^ Hep3B cells were inoculated subcutaneously into the left flank of each nude mouse. 1 week after inoculation, all mice were divided randomly into two groups (six mice per group) and treated every week with multiple-center intratumoral injection of rAd-p53 or saline per animal. The dose of rAd-p53 administered was 1×10^7^ VP/mm^3^ tumor for each group, the anticancer agents were diluted to 0.1 mL for tumors with the largest diameters of 0.5–0.9 cm, 0.2 mL for 1.0–1.4 mL tumors, and 0.3 mL for those more than 1.5 cm [16]. The tumor volume for each mouse was determined by measuring in two dimensions and calculated as tumor volume = length× (width)^2^ /2. After 4 weeks treatment, all mice were sacrificed by cervical dislocation under anesthesia with ether and the xenograft tumor tissue was explanted for routine pathological examination. Tumor tissues were subjected to immunohistochemical analysis, and a fraction was homogenized for protein extraction and immunodetection of p53 and β-actin.

### Immunohistochemistry

Tumor xenograft samples were fixed in 10% buffered formalin solution and embedded in paraffin. Fbxw7 (1:100), c-Myc (1:100) and Cyclin E (1:100) antibodies were in immunohistochemistry with streptavidin peroxidase conjugated method (SP–IHC). Immunohistochemistry was performed as previously reported [7].

### Statistical analysis

The SPSS 13.0 statistical package (SPSS, Chicago, USA) was used for all calculations. Differences between two groups were estimated with Student’s t test and ANOVA. One-way ANOVA was used for statistical comparisons among four groups. The correlation between Fbxw7 mRNA expression levels and colony formation numbers was analyzed with Linear regression and correlation analysis. The differences between groups were considered to be statistically significant when the *P* value was <0.05.

## Results

### Fbxw7 mRNA levels correlated negatively with colony formation ability of HCC cell lines

Fbxw7 is a mediator of c-Myc and Cyclin E proteolysis modulating cell cycle regulation. We measured Fbxw7 mRNA expression level and assessed colony formation ability of LO2 cells, a non transformed human liver cell line, and of the HCC cell lines SMMC-7721, Bel-7402, Hep3B, Huh7 and HepG2. Cell lines expressing the highest Fbxw7 mRNA levels showed the poorest ability to form colonies eg. LO2 and Hep3B cells (Figure 1A and 1B). Thus, Fbxw7 mRNA expression level was negatively correlated with the number of cell colonies (t=-4.124, *r* = -0.900, *P* = 0.015, Figure 1C).

**Figure 1:** Fbxw7 mRNA expression correlates negatively colony formation ability in HCC cell lines. A) The Fbxw7 mRNA expression level of HCC cell lines (n=3). B) Colony formation assay quantification with HCC cell lines. C) Correlation plot for Fbxw7 mRNA levels and colony number. Values are depicted as mean±standard error.

Fbxw7 siRNA knockdown in LO2 and Hep3B increased c-Myc and Cyclin E expression as well as cell proliferation

Since the presence of Fbxw7 reduces the ability of cell colony formation, we investigated whether the ablation of Fbxw7 mRNA affects cell proliferation and expression of cell cycle regulators as c-Myc and Cyclin E, both degradation targets of Fbxw7. We confirmed by qRT-PCR high levels of Fbxw7 mRNA in LO2 cells, and its successful knockdown by the administration of an Fbxw7 specific siRNA (Figure 2A). The Fbxw7 knockdown led to increased c-Myc and Cyclin E protein levels as shown by Western blot analysis (Figure 2B). Furthermore, we evaluated the proliferation of LO2 cells with and without Fbxw7-specific siRNA using MTT assay. The MTT activity of LO2 cells transfected with Fbxw7 siRNA was significantly increased compared control cells, suggesting higher proliferation rates (Figure 2C). The Hep3B cell line behaved similarly under Fbwx7 suppressing conditions (Figure 2A, 2B and 2C).

**Figure 2:** Effect of Fbxw7 knockdown on LO2 and Hep3B cell lines. A) qRT-PCR confirmed knockdown in LO2 and Hep3B cells treated with Fbxw7 siRNA. B) Expression of c-Myc and Cyclin E proteins were enhanced by Fbxw7 siRNA, as confirmed by Western blot analysis. β-actin served as loading control. C) Proliferation rates were assessed by MTT assay. Cell viability was normalized to time point 0 h. The proliferation rate of LO2 and Hep3B cells treated with Fbxw7 siRNA was significantly greater than in control siRNA cells. Values are depict as mean±standard error, n=3. *P<0.05 *vs* control siRNA.

### Expression of Fbxw7 is not compromised by mutations in HCC cell lines

We have previously shown decreased Fbxw7 mRNA and protein levels in HCC tumor tissues [7]. These, together with the latter in vitro results, support the model of tumor suppressive activity of Fbxw7 in HCC. It has been shown that *Fbxw7* is inactivated by mutations in diverse human cancer types with an overall mutation frequency of ~ 6% [17]. We examined *Fbxw7* cDNA derived from LO2 cell lines and HCC cell lines SMMC-7721, Bel-7402, Hep3B, Huh7 and HepG2. No mutations, such as missense mutations, deletions or insertions were detected performing database alignments, suggesting that other mechanisms might be involved in Fbxw7 inactivation contributing to an oncogenic phenotype.

### rAd-p53 decreased c-Myc and Cyclin E levels, increased Fbxw7 expression and induced apoptosis

Fbwx7 protein has been shown to be one target of the p53 tumor suppressor and mutations in this gene were detected in 27.8 to 50% of HCC cases in several studies involving patients of different ethnicities [8,18,19]. We have previously shown that Fbwx7 protein expression was negatively correlated with mutant p53 in human HCC tissues [7]. Here, we hypothesize that the exogenous expression of p53 using rAd-p53 would enhance Fbxw7 expression and thereby suppress c-Myc and Cyclin E protein expression reducing cell proliferation [20]. Initially, we performed a multiplicity of infection (MOI) gradient and MTT assay to determine the half-maximal inhibitory concentration (IC_50_) of the vector in Hep3B (Figure 3A). The p53 null cell line Hep3B was infected with rAd-p53 at an MOI of 723 (IC_50_ of rAd-p53). 48 hour after infection, p53 and Fbxw7 mRNA levels were significantly elevated compared to uninfected controls, whereas c-Myc and Cyclin E levels were slightly decreased, however not statistically significant (Figure 3B). We confirmed that rAd-p53 increased p53 and Fbwx7 protein levels not only in Hep3B cells but in HepG2 (wild type-p53) and Huh7 (mutant-p53) cells as well. In contrast, c-Myc and Cyclin E protein levels were significantly down-regulated in all three cell lines (Figure 3C). We next evaluated proliferation and apoptosis of infected Hep3B by MTT assay and flow cytometry. The proliferation of infected Hep3B cells was significantly decreased compared to uninfected control cells confirming our hypothesis (*P*<0.05, Figure 3D). Consistent with this result, 54% of Hep3B cells were AnnexinV positive and Propidium Iodide (PI) negative at 72 hours post infection (h.p.i.), indicating a significantly increase in apoptotic cells (*P*<0.05, Figure 3E).

**Figure 3:** rAd-p53 induces apoptosis in HCC cell lines with increased Fbxw7 and decreased c-Myc and Cyclin E. A) MTT activity was measured after infecting Hep3B cells with rAd-p53 in an MOI gradient to determine their IC_50_ after 48 h. Mean OD values were used to calculate the IC_50_ via the modified Kou-type method: lgIC_50_ = Xm-I (P-(3-Pm-Pn)/4), in which Xm: lg maximum dose; I: lg (maximum dose/ adjacent dose); P: sum of positive response rate; Pm: the largest positive response rate; Pn: the smallest positive response rate. B) Over-expression of *p53* 24 h after infection as confirmed by RT-PCR. Quantification of RT-PCR for p53 and Fbxw7 indicated elevated mRNA levels for rAd-p53 infected Hep3B cells, whereas c-Myc and Cyclin E levels were not significantly decreased. C) Protein expression of p53 and Fbxw7 was enhanced, while c-Myc and Cyclin E expression was suppressed by rAd-p53 in Hep3B, HepG2 and Huh7 cells, as confirmed by Western blot analysis. β-actin served as loading control. D) Hep3B proliferation rate assessed by MTT assay was significantly lower in rAd-p53 infected cells compared to control cells. E) Quantification of apoptotic cell population (AnnexinV positive/ PI negative) by flow cytometry. rAd-P53 infected Hep3B cells were composed of a larger subset of apoptotic cells after 72 hours of infection compared to control. Values are depicted as mean±standard error, n=3. *P<0.05 *vs* control.

### rAd-p53 induced apoptosis can be reverted by an Fbxw7-specific siRNA

To determine whether Fbxw7-mediated c-Myc and Cyclin E degradation participate in rAd-p53 induced apoptosis in Hep3B cells, we infected with rAd-p53 at an MOI of 723 overnight, and subsequently transfected with an Fbxw7-specific siRNA. Fbxw7 knockdown in infected Hep3B cells reverted partially the effect of exogenous p53 overexpression (Figure 4A), leading to a significant two-fold reduction of apoptotic cells and increased proliferation rates (*P*<0.05, Figure 4B and 4C). *In vitro*, these results indicate that p53 induced growth arrest and apoptosis is somewhat mediated by Fbwx7 degradation of c-Myc and Cyclin E in Hep3B cells.

**Figure 4:** rAd-p53 induced apoptosis was reverted by Fbxw7-specific siRNA. A) Fbxw7-siRNA treatment in Hep3B successfully down-regulated Fbxw7 protein but enhanced c-Myc and Cyclin expression as shown by immunostaining. Over-expression of rAd-p53 in the same cell line could enhance the levels of Fbxw7 and decrease c-Myc and Cyclin E expression. Fbxw7 knockdown in p53 over-expressing cells rescued partially the phenotype showing lower Fbxw7 levels with higher c-Myc and Cyclin E expression. β-actin served as loading control. B) The proliferation rate of rAd-p53 infected Hep3B cells was increased in the presence of Fbxw7-specific siRNA (MTT assay). C) The percentage of apoptotic Hep3B cells infected with rAd-p53 was decreased by Fbxw7-specific siRNA. Values are mean±standard error, n=3. * *P*<0.05 *vs* control; ** *P*<0.05 *vs* Fbxw7 siRNA; *** *P*<0.05 *vs* rAd-p53.

### rAd-p53 inhibits tumor growth by p53-Fbxw7 pathway *in vivo*

We next sought to determine, whether exogenous p53 affected tumor growth in Hep3B subcutaneous tumor model. Tumor bearing mice treated with 1x10^7^ rAd-p53 VP/mm3 administered by multi-center intratumoral injection, showed 2.1 fold reduction in tumor volume and 2.3 fold reduction in tumor weight compared to controls (*P*<0.05, Figure 5). We confirmed the increased expression of p53 by Western blot (Figure 6A) and performed immunohistochemistry for Fbxw7, c-Myc and Cyclin E. We could not detect c-Myc or Cyclin E in rAd-p53 treated xenografts, whereas saline treated mice showed faint Fbwx7 staining but strong c-Myc and Cyclin E signal (Figure 6B), confirming our *in vitro* observations.

**Figure 5:** rAd-p53 inhibits tumor growth *in vivo*. Multicenter intratumoral administration of rAd-P53 in Hep3B subcutaneous tumor in nude mice was monitored over time. Tumor size and weight was plotted in A), and B) respectively. C) Exemplarily, tumor bearing mice and explanted tumors are depicted. Values are mean±standard error. * *P*<0.05 *vs* rAd-p53.

**Figure 6:** p53-Fbxw7 pathway involvement in rAd-p53 treated tumor bearing mice. A) Immonostaining of tissue homogenates confirm p53 over-expression in rAd-p53 treated mice, n=3. β-actin served as loading control. B) Fbxw7, c-Myc and Cyclin E were detected by SP–IHC on paraffin sections of both groups. Tumors treated with rAd-p53 showed strong signal for Fbsw7 protein (a), while c-Myc and Cyclin E were not detectable in the same tissue section (b and c). In saline treated tumors, weak Fbxw7 staining (d) with strong c-Myc and Cyclin E staining (e and f) was detected. Micrographs were acquired at 400 fold magnification, n=6.

## Discussion

In this study, we first demonstrated that Fbxw7 is a key tumor suppressor that regulated cell proliferation in different HCC cell lines, given that Fbxw7 mRNA expression correlated negatively with colony formation ability. Ablation of Fbxw7 by RNAi in Hep3B and LO2, cell lines with high expression of the target gene, consistently showed accumulation of c-Myc and Cyclin E and enhanced cell proliferation. c-Myc protein plays crucial roles in mitogenic signaling and cell growth responses [13] and Cyclin E is a key component of the cell cycle machinery [14]. Both are frequently deregulated in HCC. This observation been reported for cell lines derived from gastric, colorectal, ovarian and breast cancer [21–24]. Here, we found a similar effect on HCC cell lines. Active Cyclin E-Cdk2 complex is required for G1-S phase transition, modulating pRb and thereby activating E2F transcription factors that enable DNA replication [25]. High levels of Fbxw7 might decrease the pool of available Cyclin E triggering arrest in G1 phase accounting for low proliferation rates. The regulation of Fbxw7 in HCC has not been yet clarified. In T-cell actue lymphoblastic leukemia (T-ALL), colorectal, breast and gastric cancer, abnormal levels of Fbxw7 have been associated with genomic mutations [22,24,26,27]. In the HCC cell lines here studied, we failed to identify any mutations, suggesting the involvement of further regulating factors. It has been shown that Fbxw7 is directly regulated by p53 [4]. Here, we showed over-expression of p53 using the commercial gene therapy drug Gendicine, which resulted in upregulation of Fbxw7 thereby preventing c-Myc and Cyclin E accumulation *in vitro* and *in vivo*. This and the observed increase in apoptosis and decrease in proliferation *in vitro*, could be partially reverted by treatment with a Fbxw7-specific siRNA. p53 is a key trigger of the intrinsic apoptotic pathway [28]. Although the levels of p53 remain unchanged in infected cells treated with Fbxw7 siRNA, a 2-fold reduction in apoptosis is observed, indicating a possible involvement of Fbxw7. We suggest that this protein contributes to trigger apoptosis during rAd-p53 administration likely by downstream effects of c-Myc degradation or unknown apoptotic effects of Fbxw7 or downstream targets. Alternatively, it has been shown that c-Myc can induce apoptosis by Caspase-3 dependent and caspase-independent signaling [29]. This mechanism might account for the significantly reduced tumor burden in Hep3B tumor model. Low proliferation rates and increase in apoptosis suggest that rAd-p53 has an anti-tumor effect as well in HCC. Intraepithelial delivery of p53 via adenoviral vectors has shown to increase apoptosis in oral leukoplakia, a well recognized precancerous lesion for squamous cell carcinoma [20].

In conclusion, we demonstrated that Fbxw7 can be activated by adenoviral delivery of p53, leading to increase proteasomal degradation of c-Myc and Cylin E. Low levels of the studied cell cycle regulators might attenuate the oncogenic phenotype of HCC cell lines by restricting G1-S transition and c-Myc mediated cell cycle reentry. Moreover, we suggest that Fbxw7 synergizes with p53 to trigger apoptosis *in vitro*. Altogether, we hypothesize that p53 contributes to hepatocarcinogenesis in part through downregulation of Fbxw7 activity and accumulation of c-Myc and Cyclin E. Addressing this pathway, we identified that rAd-p53 could be a potential therapeutic agent for HCC. Whether Fbxw7 itself is a druggable target in HCC, needs still to be clarified.
